The article "Functional activation of proline-rich tyrosine kinase2 (PYK2) in peripheral blood mononuclear cells from patients with systemic lupus erythematosus" was retracted in 2015. Reasons: duplicate publication; overlap with earlier publications.

# Functional activation of proline-rich tyrosine kinase2 (PYK2) in peripheral blood mononuclear cells from patients with systemic lupus erythematosus

**DOI:** 10.1186/1471-2474-10-141

**Published:** 2009-11-17

**Authors:** Meiying Wang, Hongsheng Sun, Wei Zhang, Yuanchao Zhang

**Affiliations:** 1 Department of Rheumatology and Immunology, Provincial Hospital affiliated to Shandong University, Jinan, 250021, China; 2 Department of Pain Management, Hospital affiliated to Medical College of Qingdao University, Qingdao, 266003, China

## Abstract

**Background:**

Systemic lupus erythematosus (SLE) is a representative systemic autoimmune disease characterized by activated T cells and polyclonally activated B cells that produce autoantibodies. Activation of autoreactive T and B cells plays a pivotal role in the pathogenesis of this disease. A role of focal adhesion kinase (FAK) in the pathogenesis has been suggested. Proline-rich tyrosine kinase2 (PYK2) is structurally related to FAK, however, the functional activation of PYK2 in SLE remains unclear. In the present study, we showed that PYK2 is significantly increased and activated in peripheral blood mononuclear cells (PBMCs) of patients with SLE. In addition, we showed the involvement of PYK2 proteins in the up-regulation of CD40L and CTLA4 expression and PBMC proliferation.

**Methods:**

Freshly isolated PBMCs from 48 SLE patients, 32 patients with rheumatoid arthritis(RA) and 24 healthy individuals were analyzed for the expression and activation of PYK2 by western-blotting and immunocytochemistry. The other isolated PBMCs from patients with this condition were cultured and stimulated with PMA or TyrA9, and then the expression of costimulatory molecules CD40L and CTLA4 was evaluated using flow cytometry, PBMCs proliferation was determined with [^3^H]-thymidine incorporation (CPM).

**Results:**

Compared with RA patients and healthy donors, PBMCs from SLE patients expressed more of both the total PYK2 protein and its activated/phosphorylated form. The increase of activated PYK2 protein in SLE PBMCs was correlated with the complication of nephritis and inversly associated the level of serum complements. In active SLE patients, activation of PYK2 in PBMCs is accompanying the increased cell proliferation and the induced expression of costimulatory molecules CD40L and CTLA4.

**Conclusion:**

Our findings indicate that phosphorylated PYK2 in SLE PBMCs may induce the expression of CD40L and CTLA4, and subsequently the cell proliferation. PYK2 signaling enhances the autoreactive lymphocyte activation and plays an important role in the pathogenesis of SLE.

## Background

Systemic lupus erythematosus (SLE) is a representative systemic autoimmune disease characterized by activated T cells and polyclonally activated B cells that produce autoantibodies. Activation of autoreactive T and B cells plays a pivotal role in the pathogenesis of this disease [1,2]. Although SLE T cells have impaired interleukin-2 (IL-2) production and proliferative response to stimulation of the T cell receptor-CD3 compound[3,4], expression of costimulatory molecules such as CD40L and CTLA4, which is essential for lymphocyte activation [5,6], is up-regulated [7-10]. These molecules are thus targets in considering effective strategies in the treatment of SLE. Lupus mice treated with antibody against CD40L or CTLA4-Ig have lower level of anti-doublestranded DNA antibodies, later development of nephritis, and prolonged survival time [11-13]. In patients with SLE, the reduced expression of CD28 costimulatory molecule on both CD4- and CD8-T cells is also well documented [14,15]. CD28-mediated costimulatory activity, following the interaction of T cells with B cells, is significantly decreased in patients with SLE [14]. Thus, it seems that costimulatory signals in SLE T cells may differ from those present in normal T cells.

The article "Functional activation of proline-rich tyrosine kinase2 (PYK2) in peripheral blood mononuclear cells from patients with systemic lupus erythematosus" was retracted in 2015. Reasons: duplicate publication; overlap with earlier publications.

Lately, in SLE T cells, focal adhesion kinase (FAK) have been shown to be involved in costimulatory molecule expression and cell proliferation[16]. Similar findings regarding the involvement of FAK were also reported in other inflammation-related diseases, such as rheumatoid arthrithis (RA)[17,18], diabetes[19], chronic inflammatory bowel diseases[20] and asthma[21]. It is thus likely that FAK may represent a new molecular target for the anti-inflammatory treatment.

The proline-rich tyrosine kinase 2 (PYK2) is a nonreceptor protein tyrosine kinase that is structurally related to FAK [22]. It is also known as cell adhesion kinase-β or related adhesion focal tyrosine kinase. Unlike the ubiquitous expression of prototype FAK, PYK2 is primarily expressed in populations of neuronal and hematopoetic cells[23]. PYK2 becomes activated in response to stimulation through a number of receptors, of which include integrins[24,25], cytokine receptors [26-28] and lymphocyte antigen receptors [29-31]. Numerous studies over the years have shown that PYK2 provides important signals during the activation of lymphocytes [32-35]. However, in SLE, PYK2's expression and activation in PBMCs, as well as the functional significance of PYK2 in T cell and B cell activation, remains unclear.

In this study, we showed that PYK2 is significantly increased and activated in PBMCs of patients with active SLE. In addition, we showed the involvement of PYK2 proteins in the up-regulation of CD40L and CTLA4 expression and PBMCs proliferation.

The article "Functional activation of proline-rich tyrosine kinase2 (PYK2) in peripheral blood mononuclear cells from patients with systemic lupus erythematosus" was retracted in 2015. Reasons: duplicate publication; overlap with earlier publications.

## Methods

The study protocol was approved by the Human Ethics Review Committee of Shandong Provincial Hospital, Jinan, China. A signed consent form was obtained from each subject prior to study participation.

### Subjects

The study subjects were 24 healthy volunteers, 32 RA patients (6 men and 26 women, mean age 42.3 years [range 21-67 years]), and 48 SLE patients (7 men and 41 women, mean age 33.9 years [range 11-69 years]), of whom 12 had inactive SLE disease and 36 had active SLE disease at the time of the study. All patients fulfilled the diagnostic criteria of the American College of Rheumatology for the classification of SLE or RA [36,37]. All SLE patients were admitted to our department between 2006 and 2009, and SLE disease activity was evaluated by the SLE Disease Activity Index (SLEDAI) score[38]. Patients were classified as having inactive disease if the SLEDAI score was persistently ≤9 for at least 3 months prior to the study. Patients with active disease had a SLEDAI score of ≥10 at the time of the study. Ten patients, 9 of whom had newly diagnosed SLE, were receiving no treatment at the time of the study. Thirty-eight SLE patients were receiving low-dose steroids (≤10 mg/day prednisolone) and/or immunosuppressive agents (cyclophosphamide). None of the SLE patients were receiving prednisolone at a dosage of ≥10 mg/day. Twenty-nine patients had biopsy-proven proliferative lupus nephritis (World Health Organization [WHO] class IV [39]), 8 had WHO class II nephritis, 4 had WHO class V nephritis, 7 had WHO class I nephritis, and 6 had central nervous system (CNS) manifestations. The clinical features of patients with and without active SLE are summarized in Table 1. All enrolled patients with RA had >6 swollen joints, >6 tender joints, and an erythrocyte sedimentation rate (Westergren) of >30 mm/hour. Twenty-six RA patients were receiving low-dose steroids (≤10 mg/day prednisolone) and/or disease-modifying antirheumatic drugs (methotrexate or sulfasalazine).

**Table 1:** Clinical features of patients with active SLE and patients with inactive SLE*

Characteristic	Patients with active disease	Patients with inactive disease
	(n = 36)	(n = 12)
No. of men/no. of women	5/31	2/10
Age, mean ± SD (range) years	35 ± 14 (11--69)	36 ± 12 (16--59)
Disease duration, mean ± SD (range) months	65 ± 101 (1--260)	118 ± 98 (5--216)
Disease activity		
SLEDAI score (0--105), mean ± SD	16 ± 4	7 ± 4
Anti-dsDNA titer, mean ± SD IU/ml	597 ± 784	49 ± 56
CH50 level, mean ± SD units/ml	14 ± 11	26 ± 8
Clinical manifestation		
WHO class IV nephritis	24	5
Other than WHO class IV nephritis	12	7
CNS disease	6	0
Treatment at time of study		
None	10	0
≤10 mg/day prednisolone	28	9
Immunosuppressive agents	7	1

* Except where indicated otherwise, values are the number of patients.

The article "Functional activation of proline-rich tyrosine kinase2 (PYK2) in peripheral blood mononuclear cells from patients with systemic lupus erythematosus" was retracted in 2015. Reasons: duplicate publication; overlap with earlier publications.

### Isolation and culture of PBMCs

Peripheral blood mononuclear cells (PBMCs) from healthy volunteers, RA patients, and SLE patients were isolated from 20 ml heparinized peripheral blood by Ficoll-Paque gradient centrifugation (Invitrogen) and then washed twice with phosphate buffered saline (PBS). The viability of PBMCs was >96% as determinded by trypan blue staining, and the purity of human T and B lymphocytes isolated was >90% as tested with anti-CD3 mAb and anti-CD19 mAb by flow cytometry. The isolated PBMCs were divided into two groups: one group was used for Western blotting and Immunocytochemistry; in the other group, the PBMCs were resuspended at 1 × 10^6 ^PBMC/ml in RPMI-1640 medium supplemented with 10% bovine fetal serum, 2 mM glutamine, 100 U/ml penicillin and 100 mg/ml streptomycin, then cultured with PMA (Sigma) or TyrA9 (Calbiochem) in 24-well culture dishes in 5% CO_2 _at 37°C to be used for further testing. Control cultures without stimulants were included in each experiment.

### Western blotting

Freshly isolated PBMCs, 2 × 10^6^, were lysed in 200 μl of cold lysis buffer (1%Triton X-100, 0.5% NP-40, 150 mM NaCl, 10 mM Tris [PH 7.4], 1 mM EDTA, 1 mM EGTA, 0.2 mM Na_3_VO_4_, 10 mM NaF, 0.2 mM PMSF, and protease inhibitors mixture) and kept on ice on a shaking platform for 30 minutes. After centrifugation at 12000 rpm for 10 minutes, supernatants were transferred to a fresh tube and stored at -80°C. Protein concentrations were determined with the BCA Protein Assay Kit (Santa Cruz Biotechnology, CA, USA). From each sample preparation, 80 ug of total proteins were mixed in Laemmli loading buffer, boiled for 4 minutes, separated by 8% SDS-PAGE and then transferred to PVDF blotting membranes (Gelman, NY, USA). Membranes were blocked with the Tris buffered saline-Tween/1% bovine serum albumin/1% nonfat dry milk and incubated with rabbit polyclonal antibodies specific for PYK2 (SC-9019), phospho-PYK2 (SC-11767-R) and β-actin (SC-1616-R) (All from Santa Cruz Biotechnology, CA, USA) overnight at 4°C (diluted according to the manufacturer's instructions). Polyclonal PYK2-specific antibody was used to detect the total protein level of PYK2 while phospho-PYK2(p- PYK2) antibody which specifically recognizes PYK2 phosphorylation on tyrosine 402 to detect the activation of PYK2. β-actin was used as a loading control to assure equal amounts of protein in all lanes. After a final incubation with a 1:5000 dilution of horseradish peroxidase-conjugated secondary antibodies (Zhongshan Biotechnology, Beijing, China) for two hours at room temperature, the membranes were developed with an ECL detection system (Santa Cruz CA, USA). For reprobing, the membranes were stripped in 0.2 *M *glycine (PH 2.5)/0.05% Tween 20 at 80°C for 20 minutes.

The article "Functional activation of proline-rich tyrosine kinase2 (PYK2) in peripheral blood mononuclear cells from patients with systemic lupus erythematosus" was retracted in 2015. Reasons: duplicate publication; overlap with earlier publications.

### Immunocytochemistry

Single immunoenzyme staining was performed using the biotin-streptavidin peroxidase method with an LSAB-HRP kit according to the manufacturer's instructions. Briefly, the freshly isolated PBMCs suspensions were put on glass slides and air-dried for at least 2 h, and either stained immediately or stored at 80°C. After air drying, the cells were fixed/permeablized with cytofix/cytoperm solution for 20 min at 4°C, dried, and washed twice in PBS pH7.2 for 5 min. The cells were incubated with blocking solution (included in kit) for 5 min in a humid atmosphere prior to the addition of primary antibody specific for phospho-PYK2 (SC-11767-R). Phospho-PYK2 antibody was added at appropriate dilution (1:100) on slides and left for 30 min in a humid atmosphere at room temperature. The cells were subsequently rinsed three times for 3 min in PBS and then allowed to react for 10 min with biotinylated antirabbit antibody (kit component). After a 3-min rinse in PBS and incubation with streptavidin-horseradish peroxidase (LSAB kit) for 30 min, the cells were washed three times in PBS (3 min each). They were then developed in diaminobenzidine, and the reaction was stopped by dipping the slides in distilled water. The cells were counterstained with 1% hematoxylin and covered with coverslips, and then examined under a light microscope. Positive cells were counted under ×400 magnification in 10 randomly chosen fields by two independent observers in a blind fashion. The results from these two observers were averaged to obtain the percentages of positive cells per sample.

### Cell staining and flow cytometric analysis

The cultured PBMCs of each well in suspension were stained with PE-CD40L (TRAP1, BD Biosciences) and PE-CTLA4 (BNI3, BD Biosciences) for 15 min at 4°C in the dark, PE-IgG1κ was used as a control. After staining, the cells were washed with cold PBS and were immediately analyzed using EPICS XL-4 flow cytometry along with system software (Becton Dickinson, San Jose, CA). The PE fluorescence intensity in PBMCs were measured using an argon laser with an excitation wavelength of 488 nm and emission wavelengths of 575 nm. The PBMCs were tightly gated by volume and complexity on S forward (0°) and side-light scattering (90°) mode. At least 1 × 10^4 ^cells were analyzed for each determination.

### Proliferation assays

For assaying PBMCs proliferation by PYK2 activation, isolated human PBMCs (2 × 10^5 ^cells/well) were cultured for 24 h in 96-well flat-bottomed microtitre plates in RPMI 1640 containing 10% FCS, stimulated with PMA or TyrA9 for the indicated duration. The cultures were pulsed with [^3^H]-thymidine (1.0 μCi/well) 18 h before harvesting the cells, and [^3^H]-thymidine incorporation was measured in a Microbeta Plus liquid scintillation counter (Wallac, Gaithersburg, MD, USA). Cultures were run in triplicate, and each experiment was repeated at least three times.

The article "Functional activation of proline-rich tyrosine kinase2 (PYK2) in peripheral blood mononuclear cells from patients with systemic lupus erythematosus" was retracted in 2015. Reasons: duplicate publication; overlap with earlier publications.

### Statistical analysis

All data were expressed as mean ± standard deviation. A one-way analysis of variance (ANOVA) test was used for comparison of more than two groups. The differences between the groups were assessed with the Post-Hoc Bonferroni test. The analysis of correlations between clinical variables and levels of p-PYK2 was based on Pearson rank test. The level of significance was set to p < 0.05. The dataset was analyzed using the SPSS V 13.0 statistical package. Each experiment was repeated at least 3 times to assess reproducibility.

## Results

### PYK2 is increased and activated in PBMCs from patients with SLE

To see the expression pattern and the activation of PYK2 in PBMCs from patients with SLE, we used Western blotting to evaluate the total amount and phosphorylated form of PYK2 in freshly isolated PBMCs from the SLE patients. As controls, PBMCs from healthy donors and RA patients were collected and processed simultaneously. As show in Figure 1A (top blot), the intensity of PYK2 band in PBMCs from SLE patients was higher than those from either heathly controls or patients with RA. Quantitative analysis shows PYK2 in PBMCs from SLE, but not RA patients (0.96 ± 0.34 in RA), was significantly up-regulated (1.13 ± 0.35 and 1.28 ± 0.30) in inactive and active SLE patients, respectively, compared with that from healthy donors (0.94 ± 0.41). Consistently, while PYK2 was weakly phosphorylated on the tyrosine 402 residue in healthy donors and RA patients, a much thicker band corresponding to p-PYK2 was seen in lanes of the SLE patients as shown in Figure 1A (middle blot). This has also been further verified by quantitative analysis in which the level of p-PYK2 was significantly higher in PBMCs from SLE patients (0.97 ± 0.31 for inactive and 1.07 ± 0.33 for active), but not in PBMCs from RA patients (0.81 ± 0.34), compared with normal PBMCs (0.77 ± 0.33) (Figure 1B). The ratio of p-PYK2/PYK2 was examined and no significant difference was found between SLE patients (0.88 ± 0.19 for inactive SLE and 0.86 ± 0.20 for active SLE), RA patients (0.85 ± 0.21) and healthy donors (0.83 ± 0.18).

**Figure 1:** **Enhanced expression and activation of PYK2 in SLE patients**. (A) Representative blot of total PYK2 and p-PYK2 in PBMCs lysates proteins obtained from healthy donors (n = 24), patients with RA (n = 32), and patients with inactive (n = 12) or active (n = 36) SLE. Total proteins obtained from PBMCs lysates were examined by Western blotting analysis for PYK2 and p-PYK2 as indicated in patients and methods. Lane 1 and 2, healthy donors;Lane 3 and 4, RA patients;Lane 5 and 6, inactive SLE patients;Lane 7 and 8, active SLE patients. (B) The ratio between the optical density of specific bands and β-actin of the same sample was calculated and expressed graphically. The experiments for each sample were repeated at least three times and bars represent the mean and standard deviation of three separate experiments. Statistical comparison of all groups was made with healthy donors. The significance level was set at* = *P *< 0.05.

The article "Functional activation of proline-rich tyrosine kinase2 (PYK2) in peripheral blood mononuclear cells from patients with systemic lupus erythematosus" was retracted in 2015. Reasons: duplicate publication; overlap with earlier publications.

To identify in which sub-population of PBMCs the activated PYK2 is expressed, we immunostained phosphorylated PYK2 in PBMCs from the samples mentioned above with an antibody against p-PYK2. As observed in Figure 2, p-PYK2 (2A and 2B) was not detectable in lymphocytes from healthy donors and RA patients, whereas in lymphocytes from SLE patients, both the intensity and the proportion of p-PYK2 immunostaining were increased (2C). These data further confirmed results obtained by Western blotting.

**Figure 2:** **Expression of p-PYK2 in PBMCs from SLE patients**. Detection of p-PYK2 protein in PBMCs from healthy donors (n = 24), patients with RA (n = 32), and patients with SLE (n = 48) was performed by immunocytochemistry technique using specific anti-p-PYK2 Abs. p-PYK2 was weakly positive in PBMCs from healthy donors (A) and RA patients (B). An increase in the positive staining for p-PYK2 was observed in PBMCs from SLE patients (C). Original magnification, × 400. Experiments were repeated at least three times with similar results.

### p-PYK2 is exclusively upregulated in SLE patients with class IV lupus nephritis and negatively correlated with the level of serum complement

We next assessed the correlation between the levels of p-PYK2 and clinical manifestation of SLE. As shown in Figure 3A and 3B, the expression of p-PYK2 was markedly up-regulated in PBMCs from SLE patients with class IV lupus nephritis, whereas this up-regulation was not seen in either healthy donors or SLE patients with CNS disease or nephritis other than class IV. Next, we analyzed the correlation between the ratio of p-PYK2/PYK2 and lupus nephritis, and no correlation was found for class IV lupus nephritis (data not shown). Furthermore, PYK2 activation and serum complement level (CH50) showed a significant negative correlation (Figure 3C). However, PYK2 activation did not show a correlation with the SLEDAI score (data not show). These results suggest that up-regulation of p-PYK2 in PBMCs is likely to be correlated with class IV nephritis.

The article "Functional activation of proline-rich tyrosine kinase2 (PYK2) in peripheral blood mononuclear cells from patients with systemic lupus erythematosus" was retracted in 2015. Reasons: duplicate publication; overlap with earlier publications.

**Figure 3:** **(A) Activation of PYK2 in PBMCs from healthy donors (n = 24) and SLE patients with central nervous system (CNS) disease (n = 6), WHO class IV nephritis (n = 29), or nephritis other than WHO class IV (n = 19)**. Total proteins obtained from PBMCs lysates were examined by Western blotting analysis for p-PYK2 as indicated in patients and methods. Lane 1, healthy donors;Lane 2, SLE patients with central nervous system; Lane 3, lupus nephritis other than WHO class IV;Lane 4, lupus nephritis IV. (B) The ratio between the optical density of specific bands and β-actin of the same sample was calculated and expressed graphically. The experiments for each sample were repeated at least three times and bars represent the mean and standard deviation of three separate experiments. Statistical comparison of all groups was made with healthy donors. The significance level was set at* = *P *< 0.05. (C) Correlation between PYK2 activation in PBMCs and serum levels of CH50 in SLE patients (n = 36).

### Enhanced PYK2 phosphorylation in PBMCs in response to lymphocyte activation stimulated by PMA

In vivo, lymphocytes often receive multiple stimuli and become activated to carry out their biologic functions. To understand the molecular events during lymphocyte activation and analyze the role played by PYK2, we tested the effect of PMA on phosphorylation of PYK2. PBMCs obtained from healthy donors, RA and SLE patients were treated with PMA or medium in 24-well culture dishes in 5% CO_2 _at 37°C for 24 h, and the status of PYK2 Y402 phosphorylation was analyzed by western boltting. As show in Figure 4A, the intensity of p-PYK2 band in PBMCs stimulated by PMA was higher than those stimulated by medium (Figure 4A). Quantitative analysis shows that p-PYK2 in PBMCs stimulated by PMA, but not by medium, was significantly up-regulated in healthy control (1.10 ± 0.32 VS 0.77 ± 0.29), RA (1.12 ± 0.35 VS 0.81 ± 0.30) and SLE (1.47 ± 0.36 VS 1.08 ± 0.34) patients, respectively (Figure 4B). These results indicate that when PBMCs were stimulated by PMA, the total level of PYK2 Y402 phosphorylation is enhanced.

**Figure 4:** **Enhanced PYK2 phosphorylation in PBMCs in response to lymphocyte activation stimulated by PMA**. (A) PBMCs obtained from healthy donors (n = 24), RA patients (n = 32) and SLE patients (n = 48) were incubated in 24-well culture dishes in 5% CO_2 _at 37°C for 24 h for with no stimulation (medium), or stimulation with PMA (1 ng/ml). Lysates prepared from 2 × 106 cells were analyzed by western blotting for the expression of p-PYK2 as indicated in patients and methods. (B) p-PYK2 expressed relative to the value obtained with PMA stimulation. Bars represent the mean and standard deviation of three separate experiments. Statistical analysis: * = p < 0.05.

The article "Functional activation of proline-rich tyrosine kinase2 (PYK2) in peripheral blood mononuclear cells from patients with systemic lupus erythematosus" was retracted in 2015. Reasons: duplicate publication; overlap with earlier publications.

### p-PYK2 in PBMCs from SLE patients induces the expression of CD40L and CTLA4

To further characterize the role of p-PYK2 in lymphocyte activation, we assayed the cell surface costimulatory molecules expression by stimulating or inhibiting PYK2 phosphorylation, using PMA and PYK2 kinase inhibitor TyrA9, respectively. As expected, using PMA to stimulate PBMCs from active SLE resulted in a significant upregulation of CD40L and CTLA4, whereas this upregulation is not observed in PBMCs pretreated with chemical inhibitor of PYK2 kinase activity (Figure 5C). In PBMCs from normal individuals and RA patients, CD40L and CTLA4 expression were also significantly upregulated by stimulation with PMA. This effect, however, cannot be suppressed by administration of TyrA9 (Figure 5A, B). These results suggest that p-PYK2 acts as an important mediator in PMA-induced induction of CD40L and CTLA4 in PBMCs of SLE.

**Figure 5:** **Up-regulation of CD40L and CTLA-4 by PYK2 activation in PBMCs from patients with active SLE (C), but not those from normal individuals and RA patients (A and B)**. PBMCs were incubated for 24 h with medium, PMA (1 ng/ml) or pretreated with the PYK2 inhibitor TyrA9 (5 μM) for 1 h before the addition of PMA, and then analyzed for the expression of CD40L and CTLA4 by flow cytometric analysis. All experiments were repeated at least three times with similar results. Statistical analysis: * = p < 0.05.

### p-PYK2 promotes the proliferation of SLE PBMCs

To explore whether upregulation of p-PYK2 may contribute to the pathogenesis of SLE, we cultured PBMCs from patients with this condition as well as from those with RA and healthy controls. Cultured cells were subjected to groups in the presence or absence of TyrA9 before stimulated with PMA and the subsequent cell proliferation assay. We found in cultures without TyrA9, the proliferation of PBMCs from all sources were enhanced by PMA. However, in the presence of TyrA9, only PBMCs from SLE patients showed a repressed proliferation when stimulated with PMA (Figure 6). These results indicate p-PYK2 transduces an activation signal for cell proliferation exclusively in PBMCs of SLE.

**Figure 6:** **Induction of cells proliferation by PYK2 activation in PBMCs from patients with active SLE, but not those from normal individuals and RA patients. **Isolated human PBMCs were cultured for 24 h in 96-well flat-bottomed microtitre plates with medium, PMA (1 ng/ml) or pretreated with the PYK2 inhibitor TyrA9 (5 μM) for 1 h before the addition of PMA, and then the cultures were pulsed with [^3^H]-thymidine (1.0 μCi/well) 18 h before harvesting the cells, and [^3^H]-thymidine incorporation was measured. The mean ± SD of the counts per minute value from triplicate samples is shown. The experiments were performed more than three times, and a representative data set is presented. * = *P *< 0.05.

The article "Functional activation of proline-rich tyrosine kinase2 (PYK2) in peripheral blood mononuclear cells from patients with systemic lupus erythematosus" was retracted in 2015. Reasons: duplicate publication; overlap with earlier publications.

## Discussion

In this study, we found an upregulation of PYK2 in PBMCs of SLE patients and an activation in SLE with class IV lupus nephritis. We also found the activation is negatively correlated with the level of serum complement. By isolating and culturing the PBMCs, we verified p-PYK2 a mediator specific to SLE to induce costimulatory molecules CD40L and CTLA4, and to promote the cell proliferation. This study represents the first demonstration that PYK2 expression and activation appear exclusive in SLE PBMCs and crucial for the pathogenesis of SLE.

Lymphocyte activation is a fundamental component implicated in the production of autoantibodies in SLE patients. Understanding the precise molecular mechanism of SLE lymphocyte activation will be important to develop novel therapeutic strategies targeting reduction autoantibodies and to increase the sensitivity of current treatment modalities. PYK2, a nonreceptor protein tyrosine kinase which plays pivotal roles in the regulation of lymphocyte activation[33], has drawn our attention in considering the lymphocyte activation in SLE.

Our studies showed no detection of p-PYK2 in PBMCs of RA and healthy controls. PYK2 in SLE PBMCs is not only increased but also phosphorylated at tyrosine 402 resides. These findings suggest that upregulation and activation of PYK2 may be implicated in the pathogenesis of SLE.

PYK2 has been reported overexpressed in glomeruli but not in other tissues of human and rat crescentic glomerulonephritis, and its overexpression is closely associated with the onset of glomerulonephritis[40]. In our study, we showed a marked upregulation of p-PYK2 in PBMCs from SLE patients with class IV lupus nephritis, but not healthy donors or SLE patients with CNS disease or nephritis other than class IV. Further, we found clear negative correlation between the levels of p-PYK2 and serum CH50. It suggests that signaling pathway involving PYK2 are likely to play a role in the development and progression of nephritis.

FAK, the prototype of PYK2, mediates signaling in active SLE enhancing autoreactive T cell activation by proliferation and by upregulating the expression of costimulatory molecule CD40L[16]. PYK2 also provides important signals to T and B lymphocyte activation[33,34]. Its expression and activation, however, are not seen in PBMCs from RA patients. We explored whether the similar scenario will happen in SLE. Given that costimulatory molecules are known to be a prerequisite for lymphocyte activation, we answered this question by checking the expression of costimulatory molecules and subsequent proliferation in SLE PBMCs. In contrast to what has been observed in RA, PYK2 was shown exclusively in SLE a mediator of activation signaling of proliferation. Therefore, PYK2-mediated activation of lymphocytes is not only functionally enhanced in SLE but also a process specific to SLE. Taking into account the limitations that chemical inhibitor of Pyk2 kinase activity is almost never perfect in its specificity, in subsequent experiments, we are going to use RNA-mediated interference, Pyk2-deficient PBMCs and dominant negative Pyk2 mutants to confirm the exact function of Pyk2 in regulating SLE PBMCs proliferation.

The article "Functional activation of proline-rich tyrosine kinase2 (PYK2) in peripheral blood mononuclear cells from patients with systemic lupus erythematosus" was retracted in 2015. Reasons: duplicate publication; overlap with earlier publications.

Abnormal T and B lymphocytes activation and lymphocytes death underlie the pathology of SLE[41]. Potentially autoreactive T and B lymphocytes are removed by apoptosis during development and after completion of an immune response. Paradoxically, lupus T cells exhibit both enhanced spontaneous apoptosis and defective activation-induced cell death [42]. Increased spontaneous apoptosis has been linked to chronic lymphopenia in patients with SLE[42]. By contrast, defective activation-induced cell death (AICD) may be responsible for persistence of autoreactive T and B lymphocytes, leading to expansion of antigen-spectific T cell clones[42]. Indeed, in prototypical murine SLE models (i.e., lpr/lpr and gld/gld mice), the animals are defective in Fas and FasL, respectively, which are critical elements in T cell apoptosis. Our result demonstrate that in addition to increased phosphorylation of PYK2 in SLE PBMCs, phosphorylated PYK2 signaling could also enhances the autoreactive lymphocyte activation and proliferation (Fig.5 and Fig.6). However, the mechanism that phosphorylated PYK2 induce lymphocyte proliferation is not clear. It would be interesting to investigate whether phosphorylated PYK2 could promote lymphocyte activation and proliferation via inhibition of apoptosis or via enhanced hyperreactivity of lymphocyte.

Our results, together with those of earlier studies, demonstrate that the PBMCs from SLE patients exhibit both increased activation and enhanced activity of PYK2. We strongly propose PYK2 a major contributor to the complex autoimmune pathogenesis of SLE.

## Conclusion

In the present study, We found a significant increase of both the total PYK2 protein and its activated/phosphorylated form in PBMCs from patients with SLE, particularly those with the complication of nephritis (WHO IV). There is a clear inversly correlation between the activation of PYK2 and the level of serum complements. In active SLE patients, activation of PYK2 in PBMCs is accompanying the increased cell proliferation and the induced expression of costimulatory molecules CD40L and CTLA4. These results indicate that phosphorylated PYK2 may induce the expression of CD40L and CTLA4, and subsequently the cell proliferation. PYK2 signaling enhances the autoreactive lymphocyte activation and plays an important role in the pathogenesis of SLE.

The article "Functional activation of proline-rich tyrosine kinase2 (PYK2) in peripheral blood mononuclear cells from patients with systemic lupus erythematosus" was retracted in 2015. Reasons: duplicate publication; overlap with earlier publications.

## Abbreviations

SLE: Systemic lupus erythematosus; FAK: focal adhesion kinase; PYK2: Proline-rich tyrosine kinase2; PBMC: peripheral blood mononuclear cell; RA: rheumatoid arthritis; CPM: [^3^H]-thymidine incorporation; IL-2: interleukin-2; SLEDAI: SLE Disease Activity Index; WHO: World Health Organization; CNS: central nervous system; PBS: phosphate buffered saline

## Competing interests

Wang M and Zhang W work for Provincial Hospital affiliated to Shandong University. All authors declare that they have no competing interests

## Authors' contributions

Meiying Wang has performed all the tests, has done preclinical analyses, statistics, graphics and has partially written the manuscript. Hongsheng Sun has added and operated additional experiments at the referee's suggestion, and has revised the manuscript. Wei Zhang has corrected the manuscript and has helped to write the manuscript. Yuanchao Zhang, as the last and responsible author, has initiated this study and has controlled the work. He has written and reviewed the manuscript.

## Pre-publication history

The pre-publication history for this paper can be accessed here:

http://www.biomedcentral.com/1471-2474/10/141/prepub
